# Development of a Nomogram Model to Predict in-Hospital Survival in Patients with Multiple Trauma

This article has been retracted.

**DOI:** 10.1155/2022/7107063

**Published:** 2022-08-08

**Authors:** Lin Ling, Wenchao Zhang, Qing Peng, Jing Tong

**Affiliations:** The Second Affiliated Hospital, Department of Emergency, Hengyang Medical School, University of South China, Hengyang, Hunan, 421001, China

## Abstract

**Background:**

Herein, we purposed to establish a nomogram model capable of assessing the probability of in-hospital survival in patients with multiple trauma.

**Methods:**

Our retrospective study is associated with 286 multiple trauma patients with 21 variables from 2017 to 2021 in The Second Affiliated Hospital, Hengyang Medical School, University of South China. We performed the univariate and multivariate logistic regression analyses for investigating the risk factors of multiple trauma. Further, we constructed a novel nomogram model, and this nomogram was evaluated by a calibration plot. Based on the multivariate analysis or the nomogram prediction model, we calculated the risk score of each patient for multiple trauma. Moreover, we compared the survival probability between the high-risk score and low-risk score groups. Finally, we assessed the discrimination of the risk score by using the C-index and the time-dependent receiver operating characteristics (ROC) curve.

**Results:**

Multivariate regression analysis revealed that the age and ISS scores were the independent risk factors, while the GCS score had protective effects on in-hospital survival. The high C-index and area under the curve (AUC) of the ROC curve confirmed reasonable discrimination for the multivariate analysis and the nomogram prediction model. Further, the calibration plot indicated reasonable accuracy of the nomogram predicting 30-day and 60-day survival probabilities.

**Conclusion:**

The nomogram model established here has good predictive efficacy for in-hospital survival of patients with multiple injuries.

## 1. Introduction

In times of peace, nonwar-related trauma has become one of the great challenges endangering global public health. The number of deaths due to trauma is as high as 5.8 million cases each year, among which the proportion of multiple trauma can be as high as 65% to 72% [1]. Multiple trauma is a common type of trauma, which is associated with the threatening of life injuries not only in a single organ but also in multiple organs, with more than 16 injury severity scores (ISS) [2, 3]. Among the three major peaks of death after multiple trauma, in addition to direct death, most patients die 24 h after trauma, and half of them die from hemorrhagic shock [4]. Therefore, early prediction of outcomes in multiple trauma patients and implementation of early and effective interventions can effectively reduce the two major peaks of early and late mortality.

The current early trauma scoring system [5, 6] and hematological tests can well assess the prognosis of patients with multiple trauma [7]. Recent studies have suggested that biochemical indicators such as plasma lactate level [8], blood glucose level [9], and serum calcium ion [10] could be used for prognostic assessment of multiple trauma. With the development of bedside testing techniques, these indicators have become rapidly available and early applied in emergency medicine. However, these independent indices have shortcomings such as cumbersome calculations, too many scoring indicators, and limited predictive ability in assessing patient prognosis during the initial phase of multiple trauma.

The nomogram or the alignment diagram is developed by using the multivariate regression analysis in which various predictors are integrated and then plotted on the same panel using scaled line segments at a certain scale, facilitating prognosis assessment [11]. It transforms the complex statistical regression equations into visualizing graphs, which in turn attracts the prediction model to read. This visualizing prediction model is instinctive and easily understandable for the medical researcher and clinical practitioner [12].

This study intends to collect clinical characteristics of hospitalized patients with multiple trauma to explore which indicators have early predictive value for survival and to provide a theoretical basis for early clinical assessment of multiple trauma.

## 2. Materials and Methods

### 2.1. Study Population

A retrospective study approach was taken to include patients with multiple trauma admitted to the Second Affiliated Hospital, Hengyang Medical School, University of South China Hospital from 2017 to 2021. We screened outpatients who were diagnosed with multiple trauma with an ISS score [13] of more than 16. The patients who had incomplete medical records, abandoned medical treatment, or were lost to follow-up were excluded. All patients signed informed consent forms and gave informed consent to this review study, approved by the regulations of University of South China Hospital (ethical number: YT152648).

The inclusion criteria are as follows: (1) age not less than 18 years old; (2) multiple trauma patients; and (3) complete auxiliary examination data of various trauma sites. The exclusion criteria are as follows: patients who died on the spot or came to hospital; pregnant; and lying-in women.

### 2.2. Data Collection

Patients' demographic profiles (age and sex), physiological parameters, and rapid bedside biochemical parameters were collected within the first 24 h after admission. Physiological parameters included heart rate (HR), respiratory rate (RR), systolic blood pressure (SBP), and diastolic blood pressure (DBP). Rapid bedside biochemical parameters included blood glucose (Glu), lactate (Lac), hemoglobin (Hb), hematocrit (Hct), platelet (PLT), procalcitonin (PCT), anion gap (AG), base excess (BE), pH, arterial partial pressure of carbon dioxide (PaCO2), and arterial partial pressure of oxygen (PaO2), sodium (Na+), potassium (K+). The severity of injury and the degree of coma were calculated using the ISS trauma score and Glasgow coma scale (GCS) score [14], respectively. In-hospital outcomes and follow-up times were also recorded.

### 2.3. Statistical and Computational Analysis

We performed statistical and computational analysis by using the R language software (version 3.6.3). The considered threshold was *p* < 0.05 for taking statistically significant differences between the three groups. We divided the patients into the “alive” group and the “dead” group as well as the “training” group according to whether they survived in-hospital after trauma. We expressed the categorical variables as the frequencies and percentages, and we used the chi-squared test to compare the two groups. We used the Student's *t*-test for comparing the continuous variables with normal distribution and variance homogeneity, which are expressed as mean ± standard deviation (mean ± SD). In contrast, The Wilcoxon rank-sum test was utilized for comparing the nonnormally distributed continuous variables, which are expressed as the median and interquartile range (IQR).

For each variable, we divided the patients into two groups based on the median. The survival differences between the two groups were analyzed using R package survival with the log-rank test method. We included the significant indicators in the univariate analysis into the Cox proportional risk model for multivariate analysis using the R package survival to screen the independent predictors affecting in-hospital survival of multiple trauma. Then, we utilized the independent predictors obtained from the multivariate analysis to develop a novel nomogram model (alpha value of *p* = 0.05, 1.61% of the average residual percentage). We employed the R package rms with the Cox method to develop the nomogram. We used the R package pROC (version 1.17.0.1) for plotting the receiver operating characteristic (ROC) curve to evaluate the discrimination of in-hospital survival by the risk score obtained from the Cox proportional risk model and the nomogram model, and the final data entry method tested reduced errors to less than 1–2%, a 60–80% reduction from reported values. Further, Harrell's concordance index (C-index) and calibration plot were utilized to evaluate the performance of the developed nomogram model.

## 3. Results

### 3.1. Clinical Characteristics of Patients

We include 286 patients in this study, and the clinical characteristics are displayed in Table 1. Among these, 233 patients were alive during their hospital stay, while 53 patients were dead. The numerous variables, including sex, age, PaO2, K+, Na+, SBP, and RR, are not statistically significant between the alive group and dead group. In contrast, the scores of PaCO2, Lac, AG, PCT, Glu, HR, and ISS were significantly higher in the dead group than in the alive group at the admission time in the hospital, and the scores of BE, pH, Hct, Hb, PLT, DBP, and GCS were significantly lower in the dead group than in the survival group.

### 3.2. Prognostic Factors for in-Hospital Survival

The univariate logistic regression analysis revealed the potential risk factors, including the score of Glu, Lac, HR, PaCO2, and ISS, while the protective factors are Hb, Hct, PLT, BE, pH, and GCS scores for in-hospital survival of multiple trauma patients (Figures 1 and 2). Besides, we performed the multivariate Cox regression analyses ,and the results showed that GCS score (hazard ratio [HR] 0.74, 95% confidence interval [CI] [0.68-0.81], *p* = 1.2e^−11^), age (hazard ratio [HR] 1.04, 95% confidence interval [CI] [1.02-1.06], *p* = 6.3e^−5^), and ISS score (hazard ratio [HR] 1.03, 95% confidence interval [CI] [1.00-1.06], *p* = 0.049) were independent risk factors (Figure 3). Then, patients were classified into two groups on the basis of the calculated risk score here. Survival analysis using a log-rank test showed that a high-risk score predicted poor survival (Figure 4(a)). The AUCs of ROC curve were 0.93, 0.93, 0.80, 0.82 at 15, 30, 60 and 90 days (Figure 4(b)). Further, all patients' clinical characteristics are displayed in Figure 4(c), and it could be observed that a high-risk score was related to more death cases.

### 3.3. Nomogram Construction and Evaluation

Three independent prognostic factors were incorporated into the nomogram (Figure 5(a)). The C-index of the nomogram was 0.89 (0.86-0.92). Good discrimination was also confirmed by AUCs, with 0.92 at 15 days, 0.91 at 30 days, 0.76 at 60 days, and 0.73 at 90 days (Figure 5(b)). The calibration curves at 30 and 60 days were validated with good consistency between actual observation and the prediction by the nomogram (Figure 5(c)). Further, by grouping patients by risk score, we found that patients with high-risk scores have lower survival, which indicated the advanced performance of the nomogram (Figure 6).

## 4. Discussion

In recent years, prehospital classification scores based on triage-revised trauma score (T-RTS), Vittel criteria, mechanism/Glasgow coma scale/age/systolic blood pressure score (MGAP), and new trauma score (NTS) could be used to assess the overall mortality risk of in-hospital patients with multiple trauma [15]. Especially, the two significant factors, the MGAP score [16] and the NTS score [5], could predict the mortality risk of in-hospitalized patients with AUCs up to 0.91 and 0.90, respectively. However, the above scoring systems have drawbacks. For example, some of the physiological indicators are costly and unavailable, and too many scoring indicators lead to cumbersome calculation and poor clinical applicability. There are few good predictors or tools to better assess in-hospital survival in patients with multiple trauma early after hospital admission. In our present study, we constructed a novel nomogram model on the basis of the GCS score, age, and ISS scores for 286 patients. The three indicators were simple, easily accessible, and inexpensive and the performance was good.

The GCS score is a medical method of assessing the degree of coma in patients and is correlated with the survival of multiple trauma patients. The study of Łukasz Skrzypiec et al. showed that the higher baseline GCS score is associated with the shorter ICU stay of patients and total hospitalization lengths [17]. In another relevant study of early trauma patients, Ammar Hashmi et al. revealed that the death risk was two times higher in older people (patients aged 74 years) compared to the lower aged people (patients aged 62 years). In the elderly patient population, the higher trauma score is correlated with higher death risk, with the risk of death up to 50 times higher in elderly patients with severe trauma compared to elderly patients with mild to moderate trauma [18]. By mining the dryad database for clinical information on 3,668 patients with multiple trauma admitted to the level I trauma center of the University Hospital of Zurich from January 1, 1996, to January 1, 2013 [19], Xie T et al. revealed that the several factors, including Lac, age, and GCS score, were the independent prognostic factors in multiple trauma [20]. In this study, we screened out GCS score, age, and ISS score as independent prognostic factors for multiple trauma patients.

Our study has some drawbacks. Although the samples were included as much as possible in this study, the findings still need to be validated in a multicenter prospective study. Besides, this study collected a limited variety of clinical indicators and failed to take into account more possible risk factors. In addition, the other factor affecting the prognosis of patients with multiple trauma is the cause of injury. Different injury causes and injured organs also have important influence on the death and prognosis of patients. We would record these information in our subsequent research.

In summary, we revealed the significant independent prognostic factors, including age, GCS score, and ISS score for patients with multiple trauma. The developed nomogram model here based on these could achieve individualized prognosis prediction for patients with multiple trauma, providing a visualized and clinically applicable evaluation tool.

## Figures and Tables

**Figure 1:** The Kaplan-Meier curves of some clinical characteristics in patients with multiple trauma. (a) Age. (b) Sex. (c) Blood glucose (Glu). (d) Lactate (Lac). (e) Hemoglobin (Hb). (f) Hematocrit (Hct). (g) Platelet (PLT). (h) Procalcitonin (PCT). (i) Diastolic blood pressure (DBP). (j) Systolic blood pressure (SBP). (k) Heart rate (HR). (l) Respiratory rate (RR) for influencing the Kaplan-Meier curves of patients with multiple trauma.

**Figure 2:** Kaplan-Meier curves of some clinical characteristics in patients with multiple trauma. (a) Anion gap (AG). (b) Base excess (BE). (c) pH. (d) Arterial partial pressure of carbon dioxide (PaCO2). (e) Potassium (K+). (f) Sodium (Na+). (g) Arterial partial pressure of oxygen (PaO2). (h) Glasgow coma scale (GCS) score. (i) Injury severity score (ISS) score for influencing the Kaplan-Meier curves of patients with multiple trauma.

**Figure 3:** Forest plot based on multivariate analysis of clinical characteristics in patients with multiple trauma.

**Figure 4:** The Kaplan-Meier analysis, the time-dependent ROC analysis, and the risk score analysis for the clinical signature in patients with multiple trauma. (a) The Kaplan-Meier survival curves in the high-risk score and low-risk score groups. (b) Time-dependent ROC curves showed AUCs at 15, 30, 60, and 90 days. (c) Risk score and survival status distribution of patients with multiple trauma.

**Figure 5:** Nomogram and its performance. (a) The nomogram is based on GCS score, age, and ISS score. (b) Time-dependent ROC curve. (c) Calibration plot.

**Figure 6:** The Kaplan-Meier curves were developed based on the risk score from the nomogram.

**Table 1:** Correlation between outcome and clinicopathologic characteristics of multiple trauma patients.

Characteristic	Alive	Dead	*p*	Method
n	233	53		
Sex, *n* (%)			0.819	Chisq.test
Female	64 (22.4%)	16 (5.6%)		
Male	169 (59.1%)	37 (12.9%)		
Age, median (IQR)	52 (35, 62)	55 (45, 68)	0.088	Wilcoxon
PH, median (IQR)	7.37 (7.33, 7.4)	7.3 (7.18, 7.37)	<0.001	Wilcoxon
PO2, median (IQR)	96 (86, 104)	92 (83, 102)	0.134	Wilcoxon
PCO2, median (IQR)	35.9 (31.6, 40.1)	41.5 (33.2, 46.4)	0.001	Wilcoxon
K, median (IQR)	3.5 (3.3, 3.8)	3.6 (3.2, 3.9)	0.903	Wilcoxon
Na, median (IQR)	138 (137, 140)	138 (136, 141)	0.976	Wilcoxon
Lac, median (IQR)	2.4 (1.8, 3.7)	4.5 (2.4, 7)	<0.001	Wilcoxon
BE, median (IQR)	-4.3 (-6.5, -2.6)	-7.2 (-10.3, -3.6)	<0.001	Wilcoxon
AG, median (IQR)	11.3 (8.9, 12.9)	12.8 (9.5, 14.2)	0.015	Wilcoxon
PCT, median (IQR)	0.38 (0.05, 2.27)	1.25 (0.12, 5.68)	0.004	Wilcoxon
Glu, median (IQR)	8.4 (6.89, 10.8)	9.9 (8, 14)	0.006	Wilcoxon
Hct, median (IQR)	0.34 (0.28, 0.4)	0.29 (0.26, 0.35)	<0.001	Wilcoxon
Hb, median (IQR)	115 (93, 131)	98 (79, 116)	<0.001	Wilcoxon
PLT, median (IQR)	166 (119, 210)	142 (90, 173)	0.009	Wilcoxon
SBP, mean ± SD	121.78 ± 27.53	113.32 ± 34.81	0.056	T test
DBP, mean ± SD	74.7 ± 18.59	66.13 ± 19.56	0.003	*T* test
RR, median (IQR)	21 (18, 25)	20 (17, 28)	0.801	Wilcoxon
HR, median (IQR)	89 (77, 109)	102 (85, 121)	0.008	Wilcoxon
GCS score, median (IQR)	15 (14, 15)	4 (3, 10)	<0.001	Wilcoxon
ISS score, median (IQR)	24 (18, 32)	32 (25, 43)	<0.001	Wilcoxon

## Data Availability

The data used to support this study is available from the corresponding author upon request.
